The article "Identifying developmental trajectories of worldwide road traffic accident death rates using a latent growth mixture modeling approach" was retracted in 2021. Reasons: duplicate publication; copyright claims.

# Identifying developmental trajectories of worldwide road traffic accident death rates using a latent growth mixture modeling approach

**DOI:** 10.1371/journal.pone.0212402

**Published:** 2019-02-20

**Authors:** Masoud Salehi, Tofigh Mobaderi, Mohammadreza Mehmandar, Afsaneh Dehnad

**Affiliations:** 1 Department of Biostatistics, Iran University of Medical Sciences, Tehran, Iran; 2 Department of Traffic Operations, Amin Police University, Tehran Traffic Police, Tehran, Iran; 3 Department of Foreign Languages, Iran University of Medical Sciences, Tehran, Iran; Tongji University, CHINA

## Abstract

Road Traffic Accidents (RTA) are a major worldwide public health problem. The aim of this study was to use the growth mixture model for clustering countries on the basis of the mortality rate patterns of RTAs from 2007 to 2013. We obtained the data on RTA death rates from World Health Organization reports and Human Development Index (HDI) of United Nations Development Programme reports for the years 2007, 2010 and 2013. Simple Latent Growth Models (LGM) in 181 countries were applied to estimate overall RTA mortality rate growth trajectories and the latent growth mixture modeling utilized to cluster them. According to non-linear LGM, the overall mortality rate of RTAs showed a decrease from 2007 to 2010 followed by an increase from 2010 to 2013. The HDI covariate had a significant negative and positive effect on intercept and slope of the LGM, respectively. The extracted mixture model appeared to have seven classes with different trends in RTA mortality rates. The worldwide countries were clustered into seven classes. Further studies on each of the seven classes are suggested to provide recommendations for reducing the mortality rate of the RTAs. Additionally, increasing HDI in some countries could have a significant effect on reducing the RTA death rates.

## Introduction

Road Traffic Accidents (RTA) occur when a motor vehicle such as a car, motorcycle or bicycle collides with another vehicle, pedestrian or other objects. RTAs, known as a major public health problem, are one of the main causes of morbidity and mortality in developing as well as developed countries [1]. RTAs are ranked as the eighth leading cause of death, and the first cause of death in the age range of 15 to 29 years old [2]. More than 1.2 million people lose their lives in the road traffic accidents and between 20 and 50 million people are injured worldwide annually, and the majority of them require long-term and costly treatment [2]. Traffic accidents, apart from sorrow and suffering, cause extensive social and economic loss, absorbing approximately 3% of gross national product of most countries [3]. If the pattern of RTAs death were not changed and no interventions were applied, it would be the third leading cause of death and approximately 1.9 million people would die annually by the year 2020 [6,3]. RTAs are responsible for 90 percent of the disability-adjusted life years (DALYs) lost and 85 percent of annual fatality in the developing countries [4]. However, while RTAs and the related deaths would decrease in developed countries, a rapid increase in many developing countries is anticipated to take place [4].

The article "Identifying developmental trajectories of worldwide road traffic accident death rates using a latent growth mixture modeling approach" was retracted in 2021. Reasons: duplicate publication; copyright claims.

Due to various geographical and environmental conditions, transportation infrastructure and traffic culture, the pattern of RTA death rates appear to change in different countries worldwide [5]. This heterogeneity would be reduced by considering various multilane highway segments neighboring structure in the model such as semi-nonparametric Poisson regression model or the empirical and fully Bayes approaches to conduct different types of safety analyses of the road crash frequency data [6–8]. Considering different sources of heterogeneity was the main goal of those studies to determine the risk factors of the road crash mortality. Trend analyses of longitudinal RTAs could be improved by considering heterogeneity between different sources of variation in other type of the models.

In the last decade, the latent growth modeling (LGM) and Latent Growth Mixture Modeling (LGMM) have gained popularity in longitudinal studies and recent studies have showed that these models can better elaborate the variance in an outcome and can provide a more precise parameter estimation than traditional analysis methods[9, 10]. The information of the overall growth trajectory is often presented by the intercept and slope of a latent growth factor in the LGMs and individual trajectories [11]. LGM assumes that all cases in the sample are based on a single homogeneous population, and individual growth trajectories vary randomly around the overall mean growth trajectory. However, the assumption of homogeneity in outcome growth trajectory is not always true [11]. Neglecting the possible growth heterogeneity and focusing on the overall mean growth trajectory can result in misunderstanding and incorrect inferences about outcome growth[12]. Therefore, the LGMs have extended to LGMMs to be used for classifying and identifying subgroups with differential growth trajectories of the outcome [13]. Although a study has remarked that there are variability and heterogeneity in road traffic accidents and related death rates in Asian and North African countries, very little is known about the heterogeneity in different countries around the world [14,15]. Therefore, in this study LGM and LGMM were applied to investigate the RTA death rate trends among countries of the world in a period of seven years from 2007 to 2013 with an interval of 3 years.

The article "Identifying developmental trajectories of worldwide road traffic accident death rates using a latent growth mixture modeling approach" was retracted in 2021. Reasons: duplicate publication; copyright claims.

## Methods

In this longitudinal study, the data of global RTA mortality rates per 100,000 population by country for the years 2007, 2010 and 2013 were extracted from “Global Status Report on Road Safety” of World Health Organization (WHO) reports and were considered as the response variable[3,16]. Furthermore, the 2010 Human Development Index (HDI), reported by the United Nations Development Programme (UNDP), was considered as a time independent covariate in the LGM and LGMM [17]. Since there were not significant differences in HDI between time points, the HDI for the year 2010 is considered as the time independent variable for simplicity. The extracted data were put together to construct an excel database, which consisted of 193 countries with 12 countries excluded in the final database due to incomplete information and missing data. It was also decided to include death rate of RTAs of the countries with at least two-time reports in the study.

The statistical analysis consisted of three steps. In the first step, simple latent growth modeling was used to define the overall trajectory of death rate of RTAs over a period of seven years. The simple LGM can be written as Eq 1:

$$\begin{array}{l} y_{ti}=\eta_{0i}+\eta_{1i}\lambda_{t}+\varepsilon_{ti}\\ \eta_{0i}=\eta_{0}+\varepsilon_{0i}\\ \eta_{1i}=\eta_{1}+\varepsilon_{1i} \end{array}$$ (1)

Where *y*_*ti*_ is the *i*^*th*^ observed outcome measure at time point *t*, *λ*_*t*_ representing the factor loadings which can be specified as linear or nonlinear function of time, *ε*_*ti*_ is the error term at time *t*, and *η*_0*i*_ and *η*_1*i*_ are random coefficients. The two latent growth factors *η*_0_ and *η*_1_ are the model estimated overall mean level of the initial outcome and the average rate of outcome change over time, respectively [11].

To estimate the overall mean growth trajectory, linear and nonlinear LGMs without covariate, i.e. unconditional models, were fitted to the data. Linear and nonlinear models are different because of the amount of factor loadings. Unlike the nonlinear model, in the linear model, the factor loadings are placed in equal intervals. To choose the best overall mean trajectory model, the Akaike Information Criterion (AIC) and the Bayesian Information Criterion (BIC) were utilized [18].

In the second step, latent growth mixture models were applied to examine the possible heterogeneity of outcome growth trajectories and classify countries into optimal distinct growth trajectory subgroups. At the beginning, a single class LGM was fitted to the data and then extended to the LGMM by raising the number of classes in each level. The AIC, BIC and the bootstrap likelihood ratio test (BLRT) were used to determine the optimal number of the classes, by comparing these criteria between k and (k-1) class models[19, 20]. Smaller values of the AIC, BIC and the significance of the BLRT test of the k-class model compared to (k-1) class suggest a better fit of the k-class model. The quality of latent class membership classification was determined by Entropy statistic and the average latent class probabilities exceeded 0.8 and 0.7, respectively[21]. In the final step, the HDI covariate was included in the best fitted LGMM of the previous step to evaluate its effect on the patterns and the membership of the latent class growth trajectories. Eq 2, describe a conditional LGMM model with *k* latent classes:

$$\begin{array}{l} y_{it}^{k}=\eta_{i0}^{k}+\eta_{i1}^{k}\lambda_{t}^{k}+\varepsilon_{it}^{k}\\ \eta_{i0}^{k}=\eta_{00}^{k}+\sum_{j}\beta_{01j}^{k}x_{j}+\varepsilon_{i0}^{k}\\ \eta_{i1}^{k}=\eta_{10}^{k}+\sum_{j}\beta_{11j}^{k}x_{j}+\varepsilon_{i1}^{k} \end{array}$$ (2)

Where $y_{it}^{k}$ is the *i*^*th*^ observed outcome measure at time point *t* for latent class *k* and the slope coefficients $\beta_{01}^{k}$ and $\beta_{11}^{k}$ are the fixed effects of covariates on the latent intercept and slope growth factors [11]. The path diagram of conditional LGMM is depicted in Fig 1.

The article "Identifying developmental trajectories of worldwide road traffic accident death rates using a latent growth mixture modeling approach" was retracted in 2021. Reasons: duplicate publication; copyright claims.

**Fig 1:** Path diagram of conditional latent growth mixture model (LGMM). The y variable represents observed outcome in each time point, *ε* is the error term, and the factor loadings are placed on the arrows.

Parameter estimation was handled by maximum likelihood method with robust standard errors (MLR) and the missing data are assumed to be Missing at Random (MAR). In the MAR mechanism, the propensity for a data point to be missing is not related to the variable with missing values, but it is related to both observed covariates and observed outcomes. Therefore, an individual’s propensity for missing data on the variable y is potentially related to other variables in the analysis, but not to the unobserved values of y itself [22]. The Full Information Maximum Likelihood (FIML) approach was used to deal with missing data to fit the models. As FIML uses every pieces of information in the observed data, it is more efficient and less biased than the traditional approaches such as LISTWISE deletion or PAIRWISE deletion methods [11]. All of the statistical analysis and model fitting were performed by Mplus 6.12 software.

## Results

The results of descriptive statistics of RTA death rates and HDI are shown in Table 1.

The article "Identifying developmental trajectories of worldwide road traffic accident death rates using a latent growth mixture modeling approach" was retracted in 2021. Reasons: duplicate publication; copyright claims.

**Table 1:** Descriptive statistics of RTA death rates and HDI.

Variable (year)	N	Minimum	Maximum	Mean	Std. Deviation
RTA death rate (2007)	174	1.70	48.40	19.53	10.29
RTA death rate (2010)	178	0	41.70	15.68	8.07
RTA death rate (2013)	175	1.90	73.40	16.71	9.93
HDI (2010)	177	0.36	0.94	0.68	0.16

According to Table 1, in all over the world, the mean of RTA death rates for 2007, 2010 and 2013 were 19.53, 15.68 and 16.71 per 100,000 population, respectively; and the mean of HDI was 0.68 in 2010. In 2007, from among 181 countries, the death rates of seven countries were missing; hence, the lowest death rate of 174 countries was 1.70 and the highest was 48.40 per 100,000 population. The RTA death rates of three countries were missing in 2010; the minimum and maximum death rates of 178 countries were 0 and 41.70, respectively. The minimum death rate of 175 countries (death rates of 6 countries were missing) was 1.90 and the maximum death rate was 73.40 for 2013. The HDI data of four countries were missing; therefore, the minimum HDI of 177 countries was 0.36 and the maximum was 0.94 in 2010.

Table 2, shows the results of the fitted two unconditional and conditional LGMs in two linear and nonlinear slopes for the RTA death rates of 181 countries.

**Table 2:** Parameter estimates and fit indices of different LGMs.

Estimates/ Fit	Parameter/ Statistics	Unconditional linear LGM	Unconditional Nonlinear LGM	Conditional linear LGM	Conditional Nonlinear LGM
		Mean (SE)	Mean (SE)	Mean (SE)	Mean (SE)
Estimate	Intercept	17.26 (0.79)*	19.56 (0.77)*	41.08 (3.09)*	49.68 (2.48)*
	HDI on intercept	——-	——	-33.67 (4)*	-44.57 (3.70)*
	Slope	-0.73 (0.27)*	-3.61 (0.59)*	0.80 (1.53)	-16.06 (2.74)*
	HDI on slope	——	——	-2.18 (1.95)	18.69 (4)*
Factor Loading					
	1^st^	0	0	0	0
	2^nd^	1	1	1	1
	3^rd^	2	0.74	2	0.57
Fit Index					
	AIC	3543.85	3518.53	3467.238	3420.355
	BIC	3569.44	3547.31	3499.223	3455.539

* Significant at 0.05 level

According to Table 2, the unconditional linear LGMs showed a significant decline pattern during the study period (slope = −0.73, p<0.05) with a high initial RTA death rates at the beginning of study (Intercept = 17.26, p<0.05), while the trend was downward from 2007 to 2010 (slope = −3.61, p<0.05). On the bases of the third factor loading of this model, the pattern then showed an upward change from 2010 to 2013(slope = −3.61 × (0.74 − 1) = 0.94). In the conditional linear model, the HDI covariate had a significant negative effect on the intercept (HDI on Intercept = −33.67, p<0.05) whereas no significant effect on the slope (HDI on slope = -2.18, p>0.05) was observed and the slope of the model was constant during the study period (slope = 0.80, p>0.05). Based on the fitted conditional nonlinear LGM, the estimated average death rate of RTAs at the starting point of the study (year 2007) was 49.68 (P<0.001), with the effect of HDI of −44.57 (p<0.05) on intercept. From 2007 to 2010, the estimated slope was −16.06 (p<0.05) showing a significant decrease pattern with the effect of HDI of 18.69 (p<0.05) on the slope. Regarding the factor loadings of this model, the slope increased (Slope = −16.06(0.57−1) = 6.91), with an adjustment on HDI effect (HDI on Slope = 18.69 (0.57–1) = −8.04) from 2010 to 2013.

The article "Identifying developmental trajectories of worldwide road traffic accident death rates using a latent growth mixture modeling approach" was retracted in 2021. Reasons: duplicate publication; copyright claims.

Table 2 shows that the conditional nonlinear LGM has the best model fit criteria among different fitted models emphasizing that adding HDI covariate in these models improves the goodness of fit indices. The overall growth trajectories of the observed and estimated mean of RTA death rates in four fitted models are presented in Fig 2.

**Fig 2:** Overall growth trajectories of observed and estimated mean of RTA death rates. (a) Unconditional nonlinear LGM, the estimated line is the same as the observed line (b) Unconditional linear LGM (c) conditional nonlinear LGM (d) conditional linear LGM.

Fig 2 shows that the estimated and observed growth trajectory appear to be similar in the conditional and unconditional nonlinear models, suggesting that the nonlinear model had a better fit than the linear model.

In the next step, the LGMM was used in order to explore the heterogeneity and determine the latent subgroups with different developmental RTA death rate trajectories among countries worldwide. For each of 1-class to 8-class fitted models, the BLRT test results and goodness of fit indices are presented in Table 3.

**Table 3:** Goodness of fit indices for the fitted growth mixture models.

Model	AIC	BIC	BLRT test p-value
1-Class	3518.527	3547.314	——————
2-Class	3439.389	3477.771	< 0.001
3-class	3413.549	3461.527	< 0.001
4-class	3368.826	3429.597	< 0.001
5-class	3359.313	3429.680	0.030
6-class	3330.073	3413.234	0.036
7-class	3307.814	3410.166	< 0.001
8-class	3427.482	3520.239	0.404

According to Table 3, the non-significant results of BLRT test for 8-class model shows that this model has no better fit than the 7-class model; therefore, the process of adding more classes to the model was stopped. The lower AIC and BIC values for the 7-class LGMM compared to the other LGMM models indicates that the 7-class LGMM has the best fit on the data. Advanced model testing, showed that the 7-class model consisted of six nonlinear and one linear class trends. Due to the estimated Entropy statistic (equal to 0.917) and the average latent class probability (higher than the 0.70 for each class), classification quality for the selected model was considerably appropriate. Results of the fitted 7-class model to the data are presented in Table 4.

The article "Identifying developmental trajectories of worldwide road traffic accident death rates using a latent growth mixture modeling approach" was retracted in 2021. Reasons: duplicate publication; copyright claims.

**Table 4:** Results of the fitted 7-class unconditional growth mixture model to the RTA death rate data.

Class	Trend	Intercept (SE)	Slope (SE)	Factor loadings 2007, 2010, 2013	Number of countries (percent)
1	Non-linear	33.545 (1.751)*	0.369 (0.814)	0, 1, -7.97	8 (0.0442)
2	Non-linear	31.204 (1.061)*	-12.097 (1.139)*	0, 1, 0.04	16 (0.0884)
3	Non-linear	46.679 (1.196)*	-36.837 (1.271)*	0, 1, 0.61	2 (0.0110)
4	Non-linear	39.231 (1.073)*	-24.121 (2.196)*	0, 1, 1.08	3 (0.01657)
5	Non-linear	29.800 (1.155)*	-6.408 (1.459)*	0, 1, 0.72	35 (0.19337)
6	linear	16.107 (0.498)*	-0.273 (0.369)	0, 1, 2	67 (0.37017)
7	Non-linear	9.326 (0.819)*	-3.105 (0.456)*	0, 1, 1.07	50 (0.27624)

* Significant at 0.05 level

Table 4 shows that the nonlinear class number one has a high initial status (intercept = 33.545, P-value<0.05) and a positive non-significant change rate (slope = 0.369, P-value>0.05). The nonlinear classes, number 2, 3, 4, 5 and 7 had significant intercepts with negative slopes. Thus, the pattern showed a decrease for these classes in the first three years (2007 to 2010); however, on the bases of the estimated factor loadings, the patterns were downward and upward in the next three years (2010 to 2013). For example, in the second class the estimated intercept, slope, and third loading factor were 31.20, −12.1 and 0.04, respectively. The average RTA death rates for this class was 31.20 per 100000 in the initial status with a decrease pattern by 12.1 per 100000 population in the first three years while according to the third factor loading of this class the pattern increased by 11.62 (−12.1 × (0.04 − 1) = 11.62) per 100000 from 2010 to 2013. In the linear model of class number six, which consisted of the highest number of the countries under the study (67 countries (%37)), the intercept was 16.11 (p<0.05) and the non-significant estimated slope was −0.27 (p>0.05). The estimated mean growth trajectories of RTA death rates of seven classes are depicted in Fig 3.

**Fig 3:** Observed and estimated mean growth trajectories of RTA death rates by 7-class.

In the final step, the conditional LGMM with the 7-class fitted to the RTA death rate data by adding the HDI covariate and the obtained results are shown in Table 5. HDI had a negative effect on intercept of the classes 1, 3, 5 and 6 while it had a positive effect on intercept of the other classes; however, the HDI effect on the intercept of the classes 2, 4, 6 and 7 was not significant. Also, estimated effects of the HDI on slope of the classes, was negative for the classes 2, 4, 6 to 7 and positive for the classes 1, 3 and 5 (Table 5). Except for the classes 6 and 7, all the other estimated effects of the HDI on the slope of the classes were significant. As we can see, it is hard to interpret the results from Table 5; for example, the class 5 which included 46 countries (25 percent) had a significant intercept (intercept = 41.25, p<0.05) by adjusted negative significant HDI (HDI on intercept = -22.41, p<0.05). Moreover, the estimated slope was -23.92 (p<0.05) by adjusted HDI (HDI on slope = 30.05, p<0.05) in the first three years of the study period (until 2010) and the slope of second three years equaled 17.7 (−23.92 (0.26 − 1) = 17.7) with the adjustment on HDI (HDI on slope = 30.05(0.26 − 1) = −22.24). Fig 4 displays the estimated growth trajectories of RTA death rates of seven classes with conditional LGMM.

The article "Identifying developmental trajectories of worldwide road traffic accident death rates using a latent growth mixture modeling approach" was retracted in 2021. Reasons: duplicate publication; copyright claims.

**Fig 4:** The adjusted estimate and observed growth trajectories of RTA rates by HDI in seven classes.

**Table 5:** Results of the fitted 7-class conditional growth mixture model to the RTA death rate data.

Class	Trend	Intercept (SE)	Slope (SE)	HDI on intercept (SE)	HDI on slope (SE)	Factor loadings 2007,2010,2013	Number of countries (percent)
1	Non-linear	60.64 (11.87)*	-3.74 (1.62)*	-60.37 (12.99)*	3.75 (1.69)*	0, 1, 4.97	44 (0.243)
2	Non-linear	-11.15 (33.83)	117.97 (31.36)*	51.35 (37.53)	-146.22 (33.63)*	0, 1, 0.40	6 (0.033)
3	Non-linear	53.44 (2.29)*	-146.69 (3.97)*	-17.32 (3.03)*	271.15 (7.65)*	0, 1, 0.56	3 (0.0166)
4	Non-linear	29.64 (6.29)*	7.79 (8.93)	10.29 (8.97)	-35.58 (15.17)*	0, 1, 1.28	11 (0.061)
5	Non-linear	41.25 (3.77)*	-23.92 (7.76)*	-22.40 (8.50)*	30.05 (14.23)*	0, 1, 0.26	46 (0.254)
6	linear	18.97 (4.06)*	1.86 (3.84)	-4.72 (5.91)	-2.43 (6.47)	0, 1, 2	53 (0.293)
7	Non-linear	-2.77 (31.09)	-1.28 (15.58)	17.99 (50.16)	-2.67 (20.34)	0, 1, 1.1	18 (0.099)

* Significant at 0.05 level

According to Fig 4, the first and seventh classes show lower RTA death rates compared to other classes with a slow decreasing pattern during the study period. The third and fifth classes which had an average of 44 and 28 death per 100000 population at the starting point of the study, showed a decreasing pattern by 2010 while the pattern changed from 2010 to 2013. The second class showed an increase by 2010 followed by a decrease by 2013; however, the overall RTA death rate of this class increased. Based on Table 5, the fourth class shows a decreasing growth trajectory and the sixth class shows a constant trend over the seven years of the study period.

## Discussion and conclusion

To demonstrate the growth trajectory of RTA rates of 181 countries from 2007 to 2013, first the two linear and nonlinear LGMs with and without HDI covariate were fitted, and then the conditional and unconditional LGMM were fitted to explore the heterogeneity of growth trajectories. Among the fitted LGMs, although the linear LGM had a simple interpretation, the model fit indices showed that the nonlinear LGM and specially the conditional nonlinear LGM had a better fit than the two conditional and unconditional linear LGM. The results of the LGMM confirmed the heterogeneity by identifying 7 distinct trajectories of RTA death rates. Due to this heterogeneity, using LGMs to demonstrate overall growth trajectories is not trustworthy in this population. Therefore, it is recommended to use LGMM in addition to LGM, in such studies. Moreover, the conditional LGMM can provide information to answer the following research question: “How do covariates such as HDI influence the membership and the growth trajectory within each latent class?”.

The article "Identifying developmental trajectories of worldwide road traffic accident death rates using a latent growth mixture modeling approach" was retracted in 2021. Reasons: duplicate publication; copyright claims.

According to our findings, the global RTA rate has a nonlinear growth trajectory, which shows a decrease from 2007 to 2010 and an increase from 2010 to 2013, despite the overall decrease pattern. The decrease in 2010, could be due to the increase in the percentage of the world population and the application of the comprehensive legislation on five key road safety risk factors: Helmets, Seat-belts, Speed, Drink–driving and Child restraints [3]. However, the rapid global motorization and the rise of approximately 30 million new passenger cars in the middle income countries might be responsible for the failure to apply minimum safety standards of the united nations in most of these countries, thereby increasing the RTA death rates from 2010 to 2013 [2]. Results of the conditional nonlinear LGM with HDI covariate showed that the HDI had a negative effect on the intercepts suggesting that the countries with a lower HDI have a higher RTA rates at the initial level. Also, the positive effect of the HDI on the slope of the model indicates that the RTA rate trajectories are decreasing dramatically for countries with low HDI and slowly for countries with high HDI. Based on the effect of HDI on the intercept and slope in the conditional nonlinear LGM, it can be inferred that the countries with high HDI had a low RTA rates at the starting point of the study, suggesting that there is no more incentive to decrease the RTA death rates in these countries. On the other hand, for countries with low HDI which had a high RTA death rates at 2007, the RTA death rate is considered a major public health problem requiring intervention.

LGMM was used to classify our study population (181 country) based on the RTA death rate patterns into several subgroups. The LGMM results identified and presented seven RTA growth trajectory classes. All classes except the first and sixth class showed a significant change rate during the study period with a different initial level of RTA death rates. According to Table 4, the class number one, including Dominican Republic, Iran, Iraq, Libyan Arab Jamahiriya, Nigeria, South Africa, Thailand and Venezuela (S1 Table and S1 Fig), have a high initial status with no significant improvement. Due to poorly developed and inadequately maintained road networks, insufficient resources for enforcement of traffic laws, unsafe public transportation, unsafe vehicles, and failure to meet safety standards, these countries appear to have a higher RTA rate in the world [3]. In classes number 2 and 3, consisting of 18 countries, all countries except Cook Island from Africa, show a downward trend of RTA death rates in the first three years followed by an upward trend. This is due to a national action plan with the target to reduce fatalities by 2010; however, the required human and financial resources were not allocated appropriately and the reduction in the RTAs was not achieved [23]. The class number 4 consists of three countries, Afghanistan, Egypt and United Arab Emirates, showed a high initial RTA rates followed by a dramatic decrease pattern over the study period. Due to the poor road infrastructure, most of the fatal RTAs occur among vulnerable road users including pedestrians, cyclists and two-wheeler riders in these countries [24]. According to WHO report, the reduction in the risk of death in these countries was due to the effective interventions such as speed control, use of seatbelts, child restraints and separation of pedestrians from vehicles [24]. The class number 5, which included most of African countries and Arabian Middle East countries, Kazakhstan, Kyrgyzstan and Malaysia, showed an initial high RTA death rate, followed by a slight decline rate up to 2010 and then a gradual increase from 2010 to 2013. As mentioned before, the African countries had a national action plan to reduce the RTA death rate during the last decade, but due to the insufficient resources, no improvement was observed after 2010 [23]. In addition, driving under the influence of alcohol, use of cellphones, and improper emergency medical rescue services were reported to be responsible in some of these countries [25, 26]. The class number 6, including 67 countries, showed an intermediate RTA death rate at the initial stage of the study while no improvement was observed during the study period. The class number seven had the lowest RTA rate compared with the other classes and showed a significant decreasing pattern over the study period, and most of developed countries are placed in this class (S1 Table). This is due to sustained political obligation, appropriate strategic planning and sophisticated technologies, which should be taken into consideration by countries with poor road safety and high RTA death rates [27].

The article "Identifying developmental trajectories of worldwide road traffic accident death rates using a latent growth mixture modeling approach" was retracted in 2021. Reasons: duplicate publication; copyright claims.

In the final step, the conditional LGMM was used in order to know the effect of HDI on the pattern of death rate in different classes. Based on the results of the study, the patterns and class memberships of the subgroups of two conditional LGMM and unconditional LGMM were slightly different. Therefore, the HDI had a significant effect on the class membership and death rate growth trajectories. The results of the conditional LGMM indicate that the effect of the HDI varies in different classes due to the heterogeneity in the study participants. For example, in class 1(most of the developed countries included in this class) the HDI had a significant negative effect on intercept and positive effect on the slope suggesting that by increasing HDI, the RTA death rate decreased at the initial level and the pattern of death rate declined with a slight slope during the study period. On the other hand, for class 2 (this class includes less developed countries with high RTA death rates such as Iran, Saudi Arabia, Thailand, etc.) the HDI had a positive effect on intercept and negative effect on the slope which means by increasing HDI, the mortality rate increased in the initial level and the pattern of death rate declined with a sharper slope during the study period.

Based on the RTA death rates, countries are classified into seven groups with different patterns. To reduce the mortality rates of the RTAs, it is recommended to conduct further studies on each of the 7 groups separately. Also, the effect of HDI on decreasing the mortality rate of various classes was different; thus, increasing HDI for some countries could have a significant effect on reducing the RTA death rates. The limited number of follow-up periods (2007, 2010 and 2013), and the missing RTA death rate data are the main limitations of this study. Therefore, increasing the number of follow-ups and using different statistical methods for imputation of the missing data would increase the accuracy of the models. In addition, using second-order LGMM to explore possible heterogeneity within classes can also be valuable.

## Supporting information

S1 Fig Geographical distribution of countries based on the class number. (A) Unconditional LGMM classes (B) Conditional LGMM classes.
(TIF)

S1 Table The study data and countries classes number based on conditional and unconditional LGMM. (A) Annual Death rates (per 100000 population) of RTAs (B) Human Development Index for each country in 2010.
(RAR)
